The article "Meta-Analysis of Anesthetic Efficacy and Safety of Propofol in Craniotomy Patients" was retracted in 2023. Reasons: signs of a paper mill; suspected computer-generated content; unreliable results or conclusions; concerns about the data.

# Meta-Analysis of Anesthetic Efficacy and Safety of Propofol in Craniotomy Patients

**DOI:** 10.1155/2022/6318051

**Published:** 2022-08-18

**Authors:** Qiang Zhou, Ya'nan Han, Jun Chen

**Affiliations:** Department of Anesthesiology, Tianjin Huanhu Hospital, Tianjin 300350, China

## Abstract

The anesthetic effect and safety of propofol in craniotomy patients by meta-analysis is investigated. Relevant studies consistent with the anesthetic effect and safety of propofol in craniotomy patients are searched and screened from domestic and foreign literature databases such as Wanfang Medical Center, CNKI, VIP, and PubMed, and meta-analysis is performed by RevMan 5.2 software. Experimental results show that the recovery time, intracranial pressure, cerebral edema, partial cerebral oxygen pressure, glutamate, and MDA in the propofol group are better than those in the control group (*P* < 0.05), and the incidence of superoxide dismutase, TNF-*α*, and adr in the propofol group is better than that in the control group (*P* > 0.05). Intravenous anesthesia with propofol in patients with craniotomy has the advantage of rapid recovery, and this program can improve intracranial pressure, brain edema, and brain oxygen partial pressure and help to improve oxidative stress and inflammatory reaction.

## 1. Introduction

tMost of the patients with severe brain injury have some degree of intracranial pressure and cerebral blood flow disorder, which leads to the death of patients with severe brain injury. Clinical surgery can effectively reduce the intracranial pressure and improve the blood circulation disorder and is the first choice for the clinical treatment of patients with severe brain injury [1, 2]. Intracranial pressure (ICP) and hemodynamic stability as well as cerebral oxygen supply and demand balance are the key contents of anesthesia management under the condition of stable systemic environment in neurosurgery. It is of great significance to provide patients with good surgical conditions. Early recovery of neurological function after operation is an important item to evaluate the anesthetic effect. Therefore, anesthetics have many advantages, such as good anesthetic effect, fast recovery, and low risk of adverse reactions. Propofol is a traditional clinical intravenous general anesthesia drug, which can meet the high standard requirements of rapid onset, rapid recovery, and high safety for craniotomy patients. However, at present, there is still a great controversy over the advantages and disadvantages of the application of anesthetic drugs in craniotomy [3, 4].

The purpose of this study is to determine the anesthetic efficacy and safety of propofol in craniotomy patients using a meta-analysis. Relevant studies consistent with the anesthetic effect and safety of propofol in craniotomy patients are searched and screened from domestic and foreign literature databases such as Wanfang Medical Center, CNKI, VIP, and PubMed, and meta-analysis is performed by RevMan 5.2 software. Experimental results show that the recovery time, intracranial pressure, cerebral edema, partial cerebral oxygen pressure, glutamate, and MDA in the propofol group are better than those in the control group (*P* < 0.05), and the incidence of superoxide dismutase, TNF-*α*, and adr in the propofol group is better than that in the control group (*P* > 0.05).

The article "Meta-Analysis of Anesthetic Efficacy and Safety of Propofol in Craniotomy Patients" was retracted in 2023. Reasons: signs of a paper mill; suspected computer-generated content; unreliable results or conclusions; concerns about the data.

The rest of this paper is organized as follows.  Section 2 discusses related work, followed by data and statistical methods designed in Section 3.  Section 4 shows the experimental results, and Section 5 concludes the paper with summary and future research directions.

## 2. Related Work

Propofol, as one of the fat-soluble compounds, can be quickly absorbed by the body and eliminated in a short time. Its diffusion distribution half-life is within 3 min, which makes its application in critical surgery an obvious advantage. Propofol can promote other chloride channels to activate GABA receptor chloride complexes, then desensitize GABA receptors and inhibit the central nervous system, and finally exert hypnotic effects. Propofol is composed of anesthesia. Propofol has little impact on respiratory and circulatory functions, and can effectively control intracranial pressure and maintain stable hemodynamics. Therefore, the risk of adverse reactions is low [5].

The formation of angiogenic brain edema and cytotoxic brain edema is the main pathological mechanism of the formation of brain edema. The main reason is that traumatic brain injury can cause secondary brain swelling, leading to an increase in intracranial pressure, thus increasing cerebral venous pressure and vascular resistance, leading to a decrease in cerebral blood flow and the buffering capacity of the body to intracranial pressure, and finally leading to brain edema. After brain injury, another blood-brain barrier is damaged, resulting in an increase in cerebral microvascular permeability. It leads to blood circulation disorder, intracranial pressure rise causes abnormality, brain oxygen metabolism balance is broken, calcium overload generates a large number of oxygen free radicals, and then causes damage to the brain, leading to a series of metabolism and dysfunction [6]. The ICP and cerebral edema volume of patients in the propofol group were lower and the level of PbrO2 is higher, suggesting that propofol can effectively regulate intracranial pressure and cerebral oxygen partial pressure and reduce cerebral edema and play a role in protecting brain tissue through the above ways. The mechanism by which propofol may exert the abovementioned effects is that the intracellular calcium concentration is positively correlated with the degree of brain cell injury. Intracellular calcium overload can aggravate the damage of brain nerve cells. Propofol can inhibit the extracellular voltage dependent calcium channel from entering calcium ions, playing the role of calcium ion flow and reducing calcium overload. In this way, brain tissue and brain cell functions can be effectively protected, and a large amount of sodium and water can be effectively prevented from remaining in cells, thus effectively reducing brain edema and improving brain oxygen metabolism and intracranial pressure [7].

The article "Meta-Analysis of Anesthetic Efficacy and Safety of Propofol in Craniotomy Patients" was retracted in 2023. Reasons: signs of a paper mill; suspected computer-generated content; unreliable results or conclusions; concerns about the data.

As an important central neurotransmitter glutamate, neurons play an important role in the process of information transmission. The brain surgery cells of patients with cerebral ischemia will produce certain toxicity. Malondialdehyde is a highly toxic lipid peroxide. Abnormal increase of malondialdehyde will have toxic effects on cells. SOD is a natural oxygen free radical scavenger. It can play a positive role in promoting the scavenging of oxygen free radicals in the body, thus effectively reducing the oxidative stress response [8, 9]. The group treated with propofol had lower Glu and MDA levels and higher SOD levels, suggesting that propofol can reduce oxidative stress response and protect brain tissue by regulating the expression and synthesis of Glu, MDA, and SOD. In order to analyze its mechanism of action, propofol may be used to inhibit the expression and secretion of glutamate, promote the synthesis of SOD and MDA, weaken the toxic effects of glutamate and MDA on cells, and quickly eliminate oxygen free radicals. Meanwhile, propofol has a special ring structure, which can provide hydrogen to replace high active free radicals. Thus, the lipid peroxidation stress response can be effectively reduced, thus playing a positive role in protecting brain cells [10].

Zeng et al. [11] believed that hematoma in patients with early intracerebral hemorrhage would further expand and cause damage to normal brain anatomical structure. Early transient ischemia, coagulation dysfunction, and damage of blood-brain barrier would activate abnormal secretion and expression of inflammatory factors, and plasma IL-6 and TNF-*α* levels would increase abnormally in patients with early enlarged thrombosis. The abnormal increase of TNF-*α* is the main cause of ischemia-reperfusion injury. Therefore, inhibition of the expression of inflammatory factors can be used as a reliable therapeutic index for the surgical treatment of severe craniocerebral injury. TNF-*α* levels in the propofol group are significantly lower than those in the control group, suggesting that propofol can reduce perioperative inflammatory response and cascade stress response in craniotomy patients. It is speculated that the reason may be that propofol can inhibit the secretion of adrenocortical hormone, thereby slowing down the production of cortisol and catecholamines, inhibit the stress fan response, play the role of adrenocorticotropic hormone in reducing the perioperative stress response, and effectively regulate TNF-ɑ and the expression level of other inflammatory factors [12].

The article "Meta-Analysis of Anesthetic Efficacy and Safety of Propofol in Craniotomy Patients" was retracted in 2023. Reasons: signs of a paper mill; suspected computer-generated content; unreliable results or conclusions; concerns about the data.

## 3. Data and Statistical Methods

### 3.1. Literature Retrieval

The literature type is clinical controlled trial. Wanfang medical journal, CNKI, VIP, and PubMed conducted a meta-analysis on the anesthetic effect and safety of propofol in craniotomy patients. Studies in the last 9 years are searched. The key words are time to wake up, intracranial pressure, cerebral edema, cerebral oxygen partial pressure, glutamic acid, malondialdehyde, plasma superoxide dismutase, tumor necrosis factor-*α*, adverse reaction, time to wake up, intracranial pressure, cerebral edema, partial cerebral oxygen pressure, glutamate, malondialdehyde, plasma superoxide dismutase, adverse reactions, and so on, and a meta-analysis was conducted based on selected literature.

### 3.2. Quality Evaluation

The selected literature treatments are assessed using a modified Jadad scale with an overall score of 1–7, with 3 or below being low quality and vice versa.

### 3.3. Statistical Methods

RevMan 5.2 statistical software is used to analyze the study data. The count data are expressed as risk ratio (RR), the analysis statistics are expressed as standard mean difference (SMD), and each effect size is expressed as 95% confidence interval (CI). When the heterogeneity between studies is *P* < 0.1 and *I*^2^ ≥ 50%, which is statistically significant, the random effect model is adopted. There is no statistical significance in heterogeneity between studies when *P* > 0.1 and *I*^2^ < 50% are satisfied, and the fixed effect model is used in the meta-analysis.

## 4. Experimental Results

### 4.1. Features of Literature Retrieval

A total of 1 English and 12 Chinese studies are included in the Chinese and English database. There are 2 low-quality studies and 11 high-quality studies, and the basic characteristics and quality evaluation results of the included studies are shown in Table 1. In Table 1, ① represents time to wake up, ② represents intracranial pressure, ③ represents cerebral edema, ④ represents partial cerebral oxygen pressure, ⑤ represents glutamic acid, ⑥ represents malondialdehyde, ⑦ represents plasma superoxide dismutase, ⑧ denotes tumor necrosis factor-*α*, and ⑨ represents adverse reactions. There is no significant publication bias in the 13 included articles, as shown in Figures 1 and 2.

The article "Meta-Analysis of Anesthetic Efficacy and Safety of Propofol in Craniotomy Patients" was retracted in 2023. Reasons: signs of a paper mill; suspected computer-generated content; unreliable results or conclusions; concerns about the data.

### 4.2. Wake Up Time

Three references are included, and heterogeneity test shows that there is heterogeneity among the references (*I*^2^ = 98.0%, *P* < 0.00001). According to the random effect model analysis, the awakening time of the propofol group is shorter than that of the control group, and the difference is statistically significant after all studies are combined (RR: −2.80, 95% CI: (−3.21,−2.38), *P* < 0.00001).  Figure 3 shows the forest diagram of waking time. It is clearly evident from Figure 3 that the recovery time of propofol anesthesia is shorter.

### 4.3. Intracranial Pressure

Six studies are included, and heterogeneity test shows that there is heterogeneity among studies (*I*^2^ = 98.0%, *P*<0.00001). According to the random effect model analysis, ICP in the propofol group is lower than that in the control group, and the difference is statistically significant after all studies are combined (RR: −3.10, 95% CI: (−3.89,−2.31), *P* < 0.00001).  Figure 4 shows the forest map of intracranial pressure. It is clearly evident from Figure 4 that propofol anesthesia can reduce ICP.

### 4.4. Cerebral Edema

Three references are included, and heterogeneity test shows inter-literature heterogeneity (*I*^2^ = 75.0%, *P*=0.02). According to random effect model analysis, intracranial pressure in the propofol group is lower than that in the control group, and the difference is statistically significant after all studies are combined (RR: −6.71, 95% CI: (−7.91,−5.51), *P* < 0.00001).  Figure 5 shows the forest map of cerebral edema. It is clearly evident from Figure 5 that propofol anesthesia can relieve cerebral edema.

### 4.5. Partial Cerebral Oxygen Pressure

Five references are included, and heterogeneity test showed inter-literature heterogeneity (*I*^2^ = 10.0%, *P*=0.35). By fixed effect model analysis, cerebral oxygen partial pressure in the propofol group is higher than that in the control group, and the difference is statistically significant after all studies are combined (RR: 3.25, 95% CI: (−2.73,3.76), *P* < 0.00001).  Figure 6 shows the forest plot of cerebral oxygen partial pressure. It is clearly evident from Figure 6 that propofol anesthesia can increase cerebral oxygen partial pressure.

### 4.6. Glu

Three references are included. Heterogeneity test shows that there is heterogeneity among the references (*I*^2^ = 61.0%, *P*=0.08). According to the random effect model analysis, Glu in the propofol group is lower than that in the control group, and the difference is statistically significant after all studies are combined (RR: −0.62, 95% CI: (−0.70,−0.54), *P* < 0.00001).  Figure 7 shows the Glu forest map. It is clearly evident from Figure 7 that propofol anesthesia can reduce Glu.

The article "Meta-Analysis of Anesthetic Efficacy and Safety of Propofol in Craniotomy Patients" was retracted in 2023. Reasons: signs of a paper mill; suspected computer-generated content; unreliable results or conclusions; concerns about the data.

### 4.7. MDA

Three references are included, and heterogeneity test shows that there is heterogeneity among the references (*I*^2^ = 0.0%, *P*=0.92). According to the random effect model analysis, MDA in the propofol group is lower than that in the control group, and the difference is statistically significant after all studies are combined (RR: −0.83, 95% CI: (−1.21,−0.45), *P* < 0.0001).  Figure 8 shows the MDA forest map. It is clearly evident from Figure 8 that propofol anesthesia can reduce MDA.

### 4.8. SOD

Four references are included, and heterogeneity test shows that there is heterogeneity among the references (*I*^2^ = 99.0%, *P* < 0.00001). According to the analysis of random effect model, SOD in propofol group is higher than that in the control group, and there is no statistical significance after all studies are combined (RR: −3.31, 95% CI: (−0.96,7.57), *P*=0.13).  Figure 9 shows the SOD forest map. It is clearly evident from Figure 9 that propofol anesthesia can reduce SOD.

### 4.9. Tumor Necrosis Factor-*α*

Four references are included, and heterogeneity test shows that there is heterogeneity among the references (*I*^2^ = 99.0%, *P* < 0.00001). The TNF-*α* level in the propofol group is lower than that in the control group by random effect model analysis, and there is no statistically significant difference between the combined studies (RR: −0.02, 95% CI: (−0.10,0.07), *P*=0.72).  Figure 10 shows the tumor necrosis factor-*α* forest map. It is clearly evident from Figure 10 that propofol anesthesia can reduce TNF-*α*, but the effect is not obvious.

### 4.10. Adverse Reactions

Two references are included, and heterogeneity test shows that there is heterogeneity among the references (*I*^2^ = 21.0%, *P*=0.26). According to fixed effect model analysis, the incidence of adverse reactions in the propofol group is lower than that in the control group, and there is no statistically significant difference between the combined studies (RR: −0.10, 95% CI: (−0.22,0.02), *P*=0.10).  Figure 11 shows the forest map of adverse reactions. It is clearly evident from Figure 11 that propofol anesthesia can reduce the incidence of adverse reactions, but the effect is not obvious.

Through the above experimental results, it can be observed that the awakening time of patients in the propofol group is significantly shorter and the incidence of adverse reactions is lower, indicating that propofol has the advantages of quick onset and short awakening time.

The article "Meta-Analysis of Anesthetic Efficacy and Safety of Propofol in Craniotomy Patients" was retracted in 2023. Reasons: signs of a paper mill; suspected computer-generated content; unreliable results or conclusions; concerns about the data.

## 5. Conclusion and Future Work

The number of studies included in this study is small, and there are still insufficient indicators in the end, which may affect the overall reference value to a certain extent. The existing studies on the balance of brain oxygen supply and demand, the impact of different anesthetic effects on the clinical anesthesia of surgical patients and the impact on the overall safety can be used as a follow-up to further improve the study and analyze the design concept of the new room.

In general, propofol intravenous anesthesia in patients with surgical operation application can improve the intracranial pressure, cerebral edema, and cerebral oxygen partial pressure. Meanwhile, it can improve Glu, MDA, SOD, and TNF-*ɑ*. Propofol can protect nerve tissue and is worth popularizing.

## Figures and Tables

**Figure 1:** Overall literature publication bias.

**Figure 2:** Publication bias of single literature.

**Figure 3:** Forest diagram of waking time.

**Figure 4:** Forest map of intracranial pressure.

**Figure 5:** Forest map of cerebral edema.

**Figure 6:** Forest plot of cerebral oxygen partial pressure.

**Figure 7:** Glu forest map.

**Figure 8:** MDA forest map.

**Figure 9:** SOD forest map.

**Figure 10:** Tumor necrosis factor-*α* forest map.

**Figure 11:** Forest map of adverse reactions.

**Table 1:** Literature information and quality.

Author	Particular year	Outcome index	Quality score

Yang et al. [13]	2016	⑨	2
Necib et al. [14]	2013	①	3
Xin [15]	2018	②③	4
Ding et al. [16]	2014	②③	4
He [17]	2019	②⑧	4
Hao et al. [18]	2018	④⑤⑥⑦	5
Pan [19]	2017	④⑤⑥⑦	5
Pan [20]	2017	①④⑦⑧	5
Cai [21]	2016	⑤⑥⑦	4
Chen [22]	2015	②④	7
Li [23]	2014	①②④	5
Hu et al. [24]	2014	②③	4
Zhou et al. [25]	2018	⑧⑨	4

## Data Availability

The simulation experiment data used to support the findings of this study are available from the corresponding author upon request.
